The article "Sirtuin 1 Induces Choroidal Neovascularization and Triggers Age-Related Macular Degeneration by Promoting LCN2 through SOX9 Deacetylation" was retracted in 2024. Reasons: signs of a paper mill; compromised peer review; unreliable results or conclusions.

# Sirtuin 1 Induces Choroidal Neovascularization and Triggers Age-Related Macular Degeneration by Promoting LCN2 through SOX9 Deacetylation

**DOI:** 10.1155/2022/1671438

**Published:** 2022-06-09

**Authors:** Su Zhao, Zhi Huang, Hao Jiang, Jiangfan Xiu, Liying Zhang, Qiurong Long, Yuhan Yang, Lu Yu, Lu Lu, Hao Gu

**Affiliations:** ^1^Department of Ophthalmology, The Affiliated Hospital of Guizhou Medical University, Guiyang 550002, China; ^2^School of Clinical Medicine, Guizhou Medical University, Guiyang 550002, China; ^3^School of Basic Medical Science, Guizhou Medical University, Guiyang 550002, China; ^4^Shenzhen Key Laboratory of Ophthalmology, Shenzhen Eye Hospital, Shenzhen 5180403, China

## Abstract

Increasing studies have identified the function of sirtuin-1 (SIRT1) in ocular diseases. Hence, this study is aimed at exploring the potential role of SIRT1 in choroidal neovascularization- (CNV-) induced age-related macular degeneration (AMD) development and the associated mechanism. Expression of SIRT1/SOX9/LCN2 in the hypoxic cells was determined, and their interactions were predicted by bioinformatics websites and followed by the verification by luciferase assay and chromatin immunoprecipitation (ChIP). Their *in vitro* effects on hypoxic cells concerning cell viability, apoptosis, migration, and angiogenesis were detected through gain- and loss-of-function assays. Besides, their *in vivo* effect was explored using the established CNV mouse models. Highly expressed LCN2, SOX9, and SIRT1 were observed in hypoxic cells. LCN2 was increased by SOX9 and SIRT1 deacetylated SOX9 to promote its nuclear translocation, which further inhibited the viability of human retinal pigment epithelial cells and promoted cell apoptosis and angiogenesis as well as CNV-induced AMD formation. The relieving role of LCN2 inhibition on CNV-induced AMD without toxicity for mice was also demonstrated by *in vivo* experiments. Overall, SIRT1 promoted the formation of CNV-induced AMD through SOX9 deacetylation-caused LCN2 upregulation, representing a promising target for CNV-induced AMD management.

## 1. Introduction

Choroidal neovascularization (CNV), as the pathological process of the invasion of abnormal blood vessels into the subretinal space of the mammalian eye, is known as a feature of the age-related macular degeneration (AMD) [1]. AMD, the main cause of visual impairment and even blindness, is a multifactorial disorder involving the dysregulation of complement, lipid, inflammation-related, angiogenesis-related, and extracellular matrix-related pathways [2]. AMD has two types: dry AMD with the presence of drusen and atrophy and wet AMD with the features of edema and hemorrhage within or below the retina or retinal pigment epithelium besides drusen and atrophy [3]. Vascular endothelial growth factor inhibitor (anti-VEGF) is a well-known medical treatment for AMD; however, this therapy is inadequate for many patients and might experience a slow loss of efficacy with repeated use [4]. Hence, new approaches are expected. Therefore, this study is aimed at providing a novel therapeutic target for CNV-induced AMD management.

The article "Sirtuin 1 Induces Choroidal Neovascularization and Triggers Age-Related Macular Degeneration by Promoting LCN2 through SOX9 Deacetylation" was retracted in 2024. Reasons: signs of a paper mill; compromised peer review; unreliable results or conclusions.

Sirtuin-1 (SIRT1) can regulate a variety of cellular functions such as metabolism, inflammation, and oxidative stresses [5–7]. Meantime, SIRT1 is a key mediator in the pathogenesis of AMD [8]. More specifically, SIRT1 also serves as a therapeutic target for CNV treatment [9]. Additionally, SIRT1 can regulate the acetylation of sex determining region Y- (SRY-) box 9 (SOX9) through nuclear translocation [10]. SOX9 belongs to the SOX gene family expressed in several organisms and involved in numerous physiological processes such as sex determination and development gonad [11]. A previous study has shown the key roles of SOX9 in the progression of CNV [1]. Moreover, SOX9 together with lipocalin 2 (LCN2) has been identified to be partially correlated with the extent of tubulointerstitial fibrosis and tubular cell injury [12]. LCN2 is a member of secreted adipokines which engaged in the pathogenesis of several diseases including cancer, diabetes, obesity, and AMD [13]. Therefore, it can be hypothesized that SIRT1/SOX9/LCN2 axis may exert great functions on the progression of CNV in AMD, but their specific interactions in CNV-induced AMD remain unclear. Hence, the present study was conducted to verify the hypothesis and explore the specific mechanism among SIRT1, SOX9, and LCN2 in the development of CNV-induced AMD, which will be greatly helpful to enlarge the understanding of CNV-induced AMD and to validate a novel therapy.

## 2. Materials and Methods

### 2.1. Ethics Statement

Animal experiments were implemented in the light of the recommendations in the Guide for the Care and Use of Laboratory Animals issued by the US National Institutes of Health.

### 2.2. Bioinformatics Analysis

AMD-related mRNA expression datasets GSE29801 and GSE103060 were downloaded from the Gene Expression Omnibus database. GSE29801 contains 151 normal samples and 142 AMD samples, while GSE103060 contains 8 normal samples and 8 AMD samples. Differential analysis was conducted using R language “limma” package to identify differentially expressed genes (DEGs) in AMD with |log fold change (FC)| >1, *p* value < 0.05 as the threshold. Transcription factors of the DEGs were predicted using the KnockTF and CistromeDB databases.

The article "Sirtuin 1 Induces Choroidal Neovascularization and Triggers Age-Related Macular Degeneration by Promoting LCN2 through SOX9 Deacetylation" was retracted in 2024. Reasons: signs of a paper mill; compromised peer review; unreliable results or conclusions.

### 2.3. Cell Culture and Hypoxia Model Construction

Human retinal pigment epithelial cells (ARPE-19, Cat.#CRL-2302) and human umbilical vein endothelial cells (HUVEC, Cat.#CRL-1730) were all purchased from the American Type Culture Collection (Manassas, VA, USA) and cultured in Dulbecco's modified Eagle's medium/F12 medium containing 10% fetal bovine serum (FBS) and 1% penicillin/streptomycin at 37°C with normoxia (consisting of 21% O_2_, 5% CO_2_, and 74% N_2_). ARPE-19 cells for hypoxia model construction were cultured in an incubator under 1% O_2_, 5% CO_2_, and 94% N_2_.

### 2.4. Cell Transfection

Lentiviruses carrying short-hairpin RNA- (sh-) SOX9, sh-SIRT1, sh-LCN2, sh-negative control (NC), overexpression- (oe-) SIRT1, oe-LCN2, oe-SOX9, and oe-NC were purchased from GenePharma (Shanghai, China). ARPE-19 cells were seeded in a 6-well plate with 2 mL culture medium per well. Cell transfection was implemented upon 50% confluency. A total of 800 *μ*L fresh virus solution (multiplicity of infection (MOI) = 30) was mixed with 800 *μ*L FBS and added with Polybrene to a final concentration of 6 *μ*g/mL. After 48 h of transfection, the cells were cultured in a medium containing puromycin (1 *μ*g/mL) for 2 weeks to select stable transfected cell lines. In order to evaluate the effect of sh-SOX9, sh-SIRT1, sh-LCN2, sh-NC, oe-SIRT1, oe-LCN2, and oe-SOX9, ARPE-19 cells were cultured in 1% serum for 2 weeks and used for the subsequent experiments.

### 2.5. Western Blot Analysis

Total protein was extracted, electrophoresed, and then electroblotted to polyvinylidene fluoride membranes. The membrane was then incubated with diluted mouse anti-SIRT1 antibody (sc-8422, 1 : 500, Santa Cruz Biotechnology, Santa Cruz, CA, USA), rabbit anti-SOX9 antibody [8242, 1 : 1000, Cell Signaling Technologies (CST), Danvers, MA, USA], acetylated-Lysine (9441, 1 : 500, CST), rabbit anti-LCN2 antibody (26991-1-AP, 1 : 1000, Proteintech, Rosemont, IL, US), and rabbit anti-*β*-actin antibody (ab8227, 1 : 1000, Abcam, Cambridge, UK) overnight at 4°C as well as with horseradish peroxidase- (HRP-) labeled secondary antibody goat anti-rabbit (ab205718, 1 : 2000, Abcam) or goat anti-mouse (ab6789, 1 : 2000, Abcam) at room temperature for 1 h. Afterwards, the membrane visualized with enhanced chemiluminescence reagent (EMD Millipore, Billerica, MA, USA) and detected by ImageQuant LAS 4000 system (General Electric Co., Boston, MA, USA). ImageJ software was used to quantify the gray values of target bands, with *β*-actin used as an internal reference.

### 2.6. Enzyme-Linked Immunosorbent Assay (ELISA)

The hypoxic ARPE-19 cells were plated and treated for 24 h. The culture medium was collected, centrifuged at 1000 g for 5 min to remove particles, and the remaining was stored at -80°C until ELISA was performed. The retinal and choroid tissues were separated from CNV mice (post-laser, 21 days), homogenized in ice-cold RIPA lysis buffer (Boster) containing 1% protease inhibitor mixture and 1% phosphatase mixture, and centrifuged at 15000 g for 15 min with the supernatant harvested for detection of the content of VEGF (human DY293B and mouse DY493, R&D Systems, Minneapolis, MN, USA), tumor necrosis factor *α* (TNF-*α*, human DY210 and mouse DY410, R&D Systems), and interleukin-6 (IL-6, human DY206 and Mouse DY406, R&D Systems) utilizing ELISA Duoset system.

The article "Sirtuin 1 Induces Choroidal Neovascularization and Triggers Age-Related Macular Degeneration by Promoting LCN2 through SOX9 Deacetylation" was retracted in 2024. Reasons: signs of a paper mill; compromised peer review; unreliable results or conclusions.

### 2.7. Cell Counting Kit 8 (CCK-8) Assay

The hypoxic ARPE-19 cells were separated, resuspended, seeded into a 96-well plate at a density of 1 × 10^5^ cells/mL (100 *μ*L) and cultured overnight. CCK-8 kit (C0037, Beyotime, Shanghai, China) was used to detect cell viability, with 3 duplicated well set. Next, the cells were incubated with 10 *μ*L of CCK-8 solution for 4 h in an incubator. Finally, the optical density (OD) value at 450 nm was measured with the help of a microplate reader followed by construction of a growth curve.

### 2.8. Flow Cytometry

The hypoxic ARPE-19 cells were resuspended and seeded in a six-well plate for overnight culture. Afterwards, the corresponding treatment was performed, and Annexin-V-fluorescein isothiocyanate/propidium iodide (AV/PI staining, 556547, BD Bioscience, San Jose, CA, USA) and flow cytometry (FACSCalibur, BD company) were applied to determine the apoptosis of ARPE-19 cells. Early apoptosis (AV single positive cells) and necrosis (AV and PI double positive cells) were quantified using FlowJo software.

### 2.9. Tube Formation Experiment

Matrigel (354234, Corning Incorporated, Corning, NY, USA) was frozen and thawed at 4°C overnight. Next, 75 *μ*L Matrigel was added to each well of a pre-chilled 96-well plate and cultured at 37°C for 60 min. HUVEC suspension was added to a 96-well plate (2.5 × 10^4^ cells/well) and incubated with the corresponding conditioned medium (CM) of ARPE-19 cells for 12-24 h, and then the appropriate field of view was selected for observation and photography under a microscope.

### 2.10. Transwell Assay

After ARPE-19 cells were treated with hypoxia and other corresponding treatments, the culture medium supernatant was collected. HUVECs were cultured in serum-free medium for 12 h, harvested, and resuspended with different CMs (1 × 10^5^/mL) in the basolateral chamber. A Transwell chamber was added with 100 *μ*L of HUVEC suspension for incubation at 37°C for 24 h. The cells migrated to the basolateral chamber were fixed with 100% methanol, dyed (Sigma-Aldrich, St. Louis, MO, USA) and counted under an inverted optical microscope (Zeiss, Jena, Germany) in 5 randomly selected visual fields.

The article "Sirtuin 1 Induces Choroidal Neovascularization and Triggers Age-Related Macular Degeneration by Promoting LCN2 through SOX9 Deacetylation" was retracted in 2024. Reasons: signs of a paper mill; compromised peer review; unreliable results or conclusions.

### 2.11. Luciferase Assay

Based on the study [14], a full-length human SOX9 cDNA was synthesized according to the UCSC (http://genome.ucsc.edu) sequence and cloned into pcDNA3.1(+) vector (Promega, Madison, WI, USA) to generate pcDNA3.1-h_SOX9. The binding motif of the transcription factor SOX9 on the promoter region of human LCN2 was predicted on the website (http://cisbp.ccbr.utoronto.ca/index.php). The human LCN2 promoter region was constructed into pGL3-Basic vector (E1751, Promega) to obtain a human LCN2-wild-type (WT) recombinant vector, and the binding motif of SOX9 on LCN2 was mutated and constructed into pGL3-Basic vector (Promega) to produce a recombinant vector of human LCN2 mutant (MUT). The constructed luciferase reporter plasmids WT and MUT were cotransfected with pcDNA3.1 (empty) or pcDNA3.1-h_SOX9 into HEK-293T cells. The luciferase activity was checked using Dual Luciferase Reporter Gene Assay Kit (E1910, Promega) and SpectraMaxi3 reader multifunctional microplate reader (Molecular Devices, San Jose, CA, USA) with Renilla luciferase as the internal control.

### 2.12. Chromatin Immunoprecipitation (ChIP) Assay

When reaching 90% confluence, cells were fixed with 1% formaldehyde for 10 min to cross-link DNA and protein, which was then terminated by glycine. The precipitate was resuspended, treated with ribozyme for 20 min, sonicated into 200-1000 bp fragments with ultrasonic wave, and randomly centrifuged at 13000 g at 4°C. The supernatant was collected and divided into four tubes. One was used as input; the remaining three were incubated with positive control antibody Histone H3, NC antibody IgG, and rabbit anti-SOX9 (82630, 1: 20, CST), respectively, overnight at 4°C. The endogenous DNA-protein complexes were precipitated with magnetic beads and centrifuged with the supernatant aspirated. The nonspecific complexes were washed, and the de-cross-linking was performed overnight at 65°C. The DNA fragments were extracted and purified to recover the DNA fragments, and the expression of the LCN2 promoter was checked by PCR. Primer sequence: forward: 5′-TGCAGAAATCTTGCCAAGTG-3′ and reverse: 5′-AGGAGACCTAGGGGCATGAT-3′.

### 2.13. Mice Model of CNV Construction

Mouse models of CNV were established by the laser irradiation. Six-week-old male C57BL/6 mice (Shanghai SLAC Laboratory Animal Co., Ltd., Shanghai, China) were housed at 22-25°C in a 12 h light/dark cycle with free access to food and water. In order to induce experimental CNV, laser-induced Bruch membrane rupture was performed on the eyes of mice after isoflurane gas anesthesia. Medical sodium hyaluronate gel was added into the experimental eye, and a 2 × 2 cm cover glass was placed in front of eyes; photocoagulation was conducted with the optic disc as the center using a slit lamp (SL120, Zeiss) with a laser (power, 200 mW; spot diameter, 100 *μ*m; exposure time, 0.1 s; wavelength, 532 nm) at 1.5-2 PD from the optic disc.

The article "Sirtuin 1 Induces Choroidal Neovascularization and Triggers Age-Related Macular Degeneration by Promoting LCN2 through SOX9 Deacetylation" was retracted in 2024. Reasons: signs of a paper mill; compromised peer review; unreliable results or conclusions.

A vitreous body was injected with lentivirus or synthetic peptide immediately after laser treatment. The mice were randomly assigned and intravitreally injected with sh-NC+oe-NC, sh-SIRT1+oe-NC, sh-NC+oe-LCN2, sh-SIRT1+oe-LCN2, 2 *μ*L of LCN2 inhibitor (RGDS peptide, *n* = 8; 5000 ng/*μ*L, ab230365, Abcam), and 2 *μ*L of placebo (RGES peptide, *n* = 8, 5000 ng/*μ*L, APC038, Shanghai Apeptide Co., Ltd., Shanghai, China). Efficacy was evaluated by isolectin B4 immunofluorescence staining.

### 2.14. Immunofluorescence Staining

After fixation, the tissue sections were sealed by 0.3% Triton X-100 in PBS and 5% goat serum protein (Beyotime, Shanghai, China) for 1 h, reacted with isolectin (1 : 1000, Santa Cruz Biotechnology) at 4°C overnight, and incubated further with secondary antibody labeled with Alexa Fluor 488 or Alexa Fluor 594 (1 : 1000, Thermo Fisher Scientific Inc., Waltham, MA, USA) for 45 min. The images were captured with the help of a fluorescence microscope (Olympus, Japan) and a Leica TCS SP8 confocal laser scanning microscope (Leica TCS NT, Wetzlar, Germany). Quantification of the CNV area was performed with the help of an image analysis software.

Cells were washed with PBS, fixed with 4% formaldehyde for 15 min, treated with 0.2% Triton X-100 PBS at 4°C for 15 min, sealed with 1% BSA for 1 h, and incubated with anti-SOX9 antibody (sc-166505, 1 : 100, Santa Cruz Biotechnology). After PBS washing for 3 times, the cells were incubated with Alexa Fluor 568-labled secondary antibody (1 : 200) for 30 min, stained with DAPI, fixed, and observed under an inverted fluorescence microscope.

### 2.15. Statistical Analysis

SPSS 22.0 statistical software (IBM Corp., Armonk, NY, USA) was utilized for analysis with measurement data summarized as the mean ± standard deviation (SD). Comparison of data between two groups was performed by an unpaired *t-*test was selected for two group comparisons, while one-way analysis of variance (one-way ANOVA) for multiple groups. *p* < 0.05 was concluded statistically significant.

## 3. Results

### 3.1. LCN2 Inhibited Hypoxic Cell Viability and Promoted Cell Apoptosis and Angiogenesis

An *in vitro* cell model of hypoxia was established using ARPE-19 cells. Western blot analysis results showed that the protein expression of E-cadherin was decreased while that of N-cadherin, Snail, and Vimentin was increased in ARPE-19 cells exposed to hypoxia (Fig. S1A), demonstrating that hypoxic ARPE-19 cells have an EMT phenotype. Furthermore, elevated LCN2 was seen in hypoxia-exposed ARPE-19 cells (Figure 1(a)). The *in vitro* effect of LCN2 on AMD was then explored. Silencing efficiency of LCN2 was confirmed by Western blot analysis, with sh-LCN2#2 presenting with higher silencing efficiency (Figure 1(b)) and thus selected for follow-up experiments. As shown in Figures 1(c)–1(g), cells transfected with sh-LCN2 presented decreased expression of VEGF, TNF-*α*, and IL-6; enhanced cell viability; and decreased cell apoptosis, migration, and angiogenesis. However, transfection with oe-LCN2 led to opposite results. Altogether, LCN2 inhibited the viability of hypoxic cells and promoted cell apoptosis and angiogenesis.

The article "Sirtuin 1 Induces Choroidal Neovascularization and Triggers Age-Related Macular Degeneration by Promoting LCN2 through SOX9 Deacetylation" was retracted in 2024. Reasons: signs of a paper mill; compromised peer review; unreliable results or conclusions.

### 3.2. SOX9 Promoted the Expression of LCN2

To explore the mechanism of LCN2 in CNV-induced AMD, potential transcription factors were predicted through the KnockTF and CistromeDB databases, and AMD-related transcription factor SOX9 was obtained after the intersection analysis with the 2015 and 1334 DEGs obtained from the GSE29801 and GSE103060 datasets, respectively (Figures 2(a)–2(c)). SOX9 was elevated in the GSE29801 (Figure 2(d)) and GSE103060 (Figure 2(e)) datasets. In addition, ARPE-19 cells after hypoxia exposure also showed increased SOX9 expression (Figure 2(f)). Western blot analysis confirmed the silencing efficiency of SOX9, evidenced by decreased SOX9 protein expression in hypoxic ARPE-19 cells following transfection of sh-SOX9#1 and sh-SOX9#2, with sh-SOX9#2 exhibiting the higher silencing efficiency (Figure 2(g)). Thus, sh-SOX9#2 (sh-SOX9) was selected for follow-up experiments. ChIP-PCR data unraveled that SOX9 was enriched in the LCN2 promoter region (Figure 2(h)). The luciferase activity of LCN2-WT in hypoxic cells transfected with oe-SOX9 was increased while that of LCN2-MUT was unaffected compared with cells transfected with oe-NC (Figure 2(i)), indicating that SOX9 elevated LCN2. Moreover, the protein expression of LCN2 in hypoxic ARPE-19 cells transfected with sh-SOX9 was reduced while oe-SOX9 caused elevated LCN2 protein expression (Figure 2(j)). To conclude, SOX9 was capable of elevating LCN2.

### 3.3. SIRT1 Inhibited the Activity of Hypoxic Cells and Promoted Cell Apoptosis and Angiogenesis by Elevating the Expression of LCN2 through SOX9 Deacetylation

Previous evidence demonstrated that SIRT1 deacetylated SOX9 [15]. We further investigated whether SIRT1 could regulate LCN2 expression by promoting SOX9 nuclear translocation through SOX9 deacetylation. We found that the expression of SIRT1 was increased in hypoxia-exposed ARPE-19 cells (Figure 3(a)). The silencing efficiency of sh-SIRT1 was confirmed by Western blot analysis, as shown by decreased protein expression of SIRT1 in cells transfected with sh-SIRT1#1 or sh-SIRT1#2, among which the silencing efficiency of sh-SIRT1# 2 was higher (Figure 3(b)), so sh-SIRT1#2 (sh-SIRT1) was selected for subsequent experiments. Besides, overexpressed SIRT1 exerted no effect on the protein expression of SOX9 but decreased the protein expression of acetylated SOX9 in the nucleus, and SIRT1 silencing upregulated the expression of acetylated SOX9 in the nucleus (Figure 3(c)). Moreover, the SOX9 fluorescence in the nucleus was notably increased in response to oe-SIRT1 but decreased upon sh-SIRT1 (Figure 3(d)), indicating that SIRT1 can promote the nuclear translocation of SOX9 through deacetylation.

The article "Sirtuin 1 Induces Choroidal Neovascularization and Triggers Age-Related Macular Degeneration by Promoting LCN2 through SOX9 Deacetylation" was retracted in 2024. Reasons: signs of a paper mill; compromised peer review; unreliable results or conclusions.

Next, it was investigated whether SIRT1 can promote SOX9 nuclear translocation by deacetylating SOX9, thereby affecting the expression of LCN2. Western blot data disclosed that SIRT1 silencing decreased SIRT1 and LCN2 and increased acetylated SOX9 expression; LCN2 overexpression played the opposite role to SIRT1 silencing; and downregulation of SIRT1 and LCN2 and upregulation of acetylated SOX9 mediated by SIRT1 silencing also could be reversed by LCN2 overexpression in hypoxic ARPE-19 cells (Figure 3(e)). In summary, SIRT1 could promote nuclear translocation of SOX9 through deacetylation, thereby promoting the expression of LCN2.

Furthermore, functional assays revealed that SIRT1 silencing causes a reduction in VEGF, TNF-*α*, and IL-6 expression, an enhancement in cell viability and an attenuation in cell apoptosis, while LCN2 overexpression could reverse the above conditions in hypoxia-exposed ARPE-19 cells (Figures 3(f)–3(h)). As shown in Figures 3(i) and 3(j), migration and tube formation of HUVECs were noted to be attenuated in the presence of SIRT1 silencing, while further overexpression of LCN2 led to opposite results.

Thus, SIRT1 promoted the SOX9 nuclear translocation through the deacetylation of SOX9, thereby promoting the expression of LCN2 to inhibit the viability of hypoxic cells and promote cell apoptosis and angiogenesis.

### 3.4. SIRT1 Promoted Laser-Induced CNV Formation in Mice by Promoting LCN2 through the Deacetylation of SOX9

Next, we focused on the role of SIRT1/SOX9/LCN2 in the laser-induced CNV model in mice. At 7 days after CNV induction by laser, the mice were treated. Western blot data revealed that SIRT1 and LCN2 were notably upregulated, while acetylated SOX9 was downregulated in the choroid/RPE tissues of mice after laser treatment (Figure 4(a)). Besides, we proved that SIRT1 silencing downregulated SIRT1 and LCN2 and upregulated acetylated SOX9 in the choroid/RPE tissues of mice, which also could be reversed by LCN2 overexpression (Figure 4(b)). We also discovered that SIRT1 silencing could reduce CNV area and LCN2 overexpression could increase CNV area. And the CNV area reduced by SIRT1 silencing can be reversed by LCN2 overexpression, and the CNV area increased by LCN2 overexpression can also be reversed by SIRT1 silencing (Figures 4(c) and 4(d)). In summary, SIRT1 promoted the expression of LCN2 by deacetylating SOX9 to promote the formation of laser-induced CNV in mice.

The article "Sirtuin 1 Induces Choroidal Neovascularization and Triggers Age-Related Macular Degeneration by Promoting LCN2 through SOX9 Deacetylation" was retracted in 2024. Reasons: signs of a paper mill; compromised peer review; unreliable results or conclusions.

### 3.5. LCN2 Inhibitors Inhibited the Formation of CNV in Mice with Rare Toxicity to Tissues

In order to further explore the potential of LCN2 inhibition in the clinical treatment of CNV, LCN2 inhibitor RGDS and placebo RGES were used for follow-up studies. Western blot analysis results showed that the protein expression of LCN2 was upregulated in the choroid/RPE tissues of mice after laser treatment. Compared with the Laser+RGES group, the protein expression of LCN2 was downregulated in the choroid/RPE tissues of mice in the Laser+RGDS group (Figure 5(a)). Additionally, CNV formation in mice after laser treatment was increased. Compared with mice treated by Laser+RGES, the Laser+RGDS treatment decreased the formation of CNV in the choroid/RPE tissues (Figures 5(b) and 5(c)). Subsequently, the maximum lesion diameter of CNV and CNV/choroid ratio were higher in mice after laser treatment than those of the control mice. To sum up, RGDS can inhibit the formation of laser-induced CNV.

## 4. Discussion

CNV is the feature of late-stage AMD and the greatest contributor for irreversible central visual loss among the elderly with AMD (Wang et al., 2016, [16, 17]). The hallmark of AMD pathogenesis is the retinal pigment epithelial cell damage induced by drusen accumulation, in which oxidative stress and inflammation are the well-known molecular mechanisms [18]. A recent study has identified the crucial role of SIRT1 in ocular diseases [19]. Here, we designed to investigate the potential mechanism of SIRT1 in CNV-induced AMD, and our final results demonstrated that SIRT1 elevated LCN2 through SOX9 deacetylation, thereby enhancing cell apoptosis, migration, and angiogenesis of hypoxic cells *in vitro* and inducing CNV formation *in vivo*.

It is reported that LCN2 is capable of protecting against ocular inflammation and thus further acts as a promising target for managing ocular diseases such as uveitis and retinal degeneration [20, 21]. LCN2 has been also confirmed as a potential target for AMD treatment [22]. More importantly, the expression of LCN2 is positively correlated with the severity of CNV in AMD [23, 24]. In our study, we proved that LCN2 could prevent viability and induce apoptosis and angiogenesis in ARPE-19 cells after hypoxia.

The article "Sirtuin 1 Induces Choroidal Neovascularization and Triggers Age-Related Macular Degeneration by Promoting LCN2 through SOX9 Deacetylation" was retracted in 2024. Reasons: signs of a paper mill; compromised peer review; unreliable results or conclusions.

Additionally, we further predicted the possible target genes of LCN2 by bioinformatics analysis, and we discovered that SOX9 is an underlying regulatory gene of LCN2 in AMD-induced CNV. A promising therapeutic role of SOX9 has been also illustrated in retinal degenerative diseases [25]. Similar to our findings, another study has also observed the downregulation of SOX9 in the dorsal neural retina, which is negatively related to the dorsal choroidal vascular development [26]. In our study, we verified that SOX9 was highly expressed in AMD and hypoxia-induced ARPE-19 cells. And we also proved that SOX9 could upregulate LCN2 in ARPE-19 cells after hypoxia.

SIRT1, a member of the sirtuin gene family, has key roles in the regulation of gene expression, maintenance of chromosome architecture, and cell cycle progression [27]. It has been reported that SIRT1 has various functions, such as antioxidant, antifree radical, antiaging, metabolic regulation, and immune regulation, all of which processes are associated with hypoxia [28]. The study proved that highly expressed SIRT1 is also observed previously in the cornea of mice with diabetic dry eyes [29]. Besides, SIRT1 was also observed to be highly expressed in the anterior capsule and peripheral blood samples of patients with age-related cataract [30]. In our study, we further found that SIRT1 presented abnormally high expression in hypoxic cells.

Furthermore, SIRT1 is a well-recognized deacetylase responsible for SOX9 deacetylation, which further induces SOX9 nuclear localization in retinal pigment epithelial cells [15, 31]. The negative regulation relationship between SIRT1 and SOX9 has been validated in a recent study [10]. To further figure out the function of SIRT1 in AMD, hypoxic cells were transfected with sh-SIRT1, and the results showed that the expression of VEGF, TNF-*α*, and IL-6 was decreased, cell viability was increased, and the cell migration, apoptosis, and angiogenesis were impaired, indicating that SIRT1 silencing exerted protecting effects on AMD progression. SIRT1 has been reported to prevent the retinal degeneration and inflammation in AMD [32]. Likewise, the therapeutic role of SIRT1 silencing on neovascular AMD has been also highlighted by a prior study [33]. VEGF, TNF-*α*, and IL-6 are well-established biomarkers for hypoxia, which are increased under the condition of hypoxia [34, 35]. Particularly, the area of laser-induced CNV can be notably decreased by inhibiting VEGF [36]. Additionally, reductions in VEGF, TNF-*α*, and IL-6 are a hallmark of the retarded formation of CNV in wet AMD [37]. Hence, these findings supported the attenuating function of SIRT1 silencing in the progression of CNV-induced AMD. Further analysis revealed that SIRT1 increased the formation of CNV in mice with AMD by increasing the expression of LCN2 through deacetylation of SOX9. Taken together, the aforementioned indicated the deteriorating role of SIRT1/SOX9/LCN2 in the CNV-induced AMD.

The article "Sirtuin 1 Induces Choroidal Neovascularization and Triggers Age-Related Macular Degeneration by Promoting LCN2 through SOX9 Deacetylation" was retracted in 2024. Reasons: signs of a paper mill; compromised peer review; unreliable results or conclusions.

However, studies have shown that SIRT1 has a protective effect against disease, which is not consistent with our current research. For example, miR-138, miR-181a, and miR-181b directly inhibited SIRT1 expression and promoted apoptosis (Wang et al. 2016; [38]). SIRT1 overexpression reversed premature cell death caused by oxidative stress [39]. Activation of SIRT1 maintained retinal barrier integrity while decreasing the expression of inflammatory factors IL-8, IL-6, and MMP-9 [32]. Overall, SIRT1 plays a key role in anti-inflammatory, antiaging, and antioxidant processes, while an additional study also showed that SIRT1 expression was upregulated in AMD samples, which is consistent with our findings. These studies suggest that SIRT1 is not necessarily protective in AMD and is more likely to be two-sided. Previous studies have revealed that SIRT1 acts as a deacetylase with many downstream substrates, such as p65 NF-*κ*B [40], STAT3 [41], and CHK2 [42], SOX9 [43], and plays different roles in various biological processes mainly for deacetylation of histones and nonhistones with different mechanisms of action. Thus, the substrates regulated by SIRT1 deacetylation are all transcription factors, and the regulation of target genes by transcription factors is strongly dependent on the cellular and disease environment. The present study targets one target gene, LCN2, which is indeed positively regulated by SIRT1/SOX9 during the CNV-induced AMD. Therefore, the different genes (SOX9 and LCN2) regulated by SIRT1 and the different cells and diseases studied are the reasons why the results of SIRT1 studies differ from previous ones.

However, there are certain limitations in the current study. For instance, although we confirmed that SIRT1 deacetylation can exacerbate AMD progression by upregulating SOX9 and increasing LCN2 expression, other signaling pathways also exist in SIRT1 to alleviate AMD progression, which requires further investigation. The effects of Oe-SIRT1 or sh-SIRT1 on angiogenesis in animals have not been addressed. The effect of SIRT1/SOX9/LCN2 axis-related inhibitors, such as RGDSv, on angiogenesis in animals needs to be further demonstrated. Exploring whether SIRT1, SOX9, and LCN2 pharmacological inhibitors can improve AMD may have more clinical application. This study validates a shallow mechanism, especially in animal experiments.

The article "Sirtuin 1 Induces Choroidal Neovascularization and Triggers Age-Related Macular Degeneration by Promoting LCN2 through SOX9 Deacetylation" was retracted in 2024. Reasons: signs of a paper mill; compromised peer review; unreliable results or conclusions.

## 5. Conclusion

In summary, our evidence pointed toward that SIRT1 deacetylated SOX9 to promote its nuclear translocation, thereby increasing the expression of LCN2, further inducing the secretion of VEGF and inflammation-related factors, as well as cell apoptosis, migration, and angiogenesis, and ultimately promoting the formation of blood vessels in CNV-induced AMD (Figure 6). Thus, this study helps to deepen the clinical understanding of the pathological process of AMD occurrence and development and provides a scientific basis for the subsequent development of targeted drugs (about SIRT1/SOX9/LCN2 axis) for AMD treatment.

## Figures and Tables

**Figure 1:** LCN2 inhibits the viability of hypoxic cells and promotes cell apoptosis and angiogenesis. (a) The protein expression of LCN2 in ARPE-19 cells exposed to hypoxia determined by Western blot analysis. (b) The protein expression of LCN2 in hypoxic cells after different transfections determined by Western blot analysis. (c) The content of VEGF, TNF-*α* and IL-6 in the cell culture fluid determined by ELISA. (d) The viability of hypoxic cells after different transfections determined by CCK-8. (e) The apoptosis of hypoxic cells after different transfections determined by flow cytometry. (f) The migration of hypoxic cells after different transfections determined by Transwell. (g) The angiogenesis of hypoxic cells after different transfection determined by tube formation experiment. ^∗^*p* < 0.05, compared with control or cells transfected with sh-NC; ^#^*p* < 0.05, compared with cells transfected with oe-NC. ^∗∗^*p* < 0.01,  ^∗∗∗^*p* < 0.001, and^∗∗∗∗^*p* < 0.0001. ^##^*p* < 0.01, ^###^*p* < 0.001, and ^####^*p* < 0.0001.

**Figure 2:** SOX9 upregulates LCN2 expression. (a) A heat map of DEGs between 151 normal samples and 142 AMD samples in GSE29801 dataset. (b) A heat map of DEGs between 8 normal samples and 8 AMD samples in GSE103060 dataset. (c) Venn diagram of the intersection among 4 datasets. (d) The expression of SOX9 in GSE29801 dataset (151 normal samples and 142 AMD samples). (e) The expression of SOX9 in GSE103060 dataset. (f) The protein expression of SOX9 in control and hypoxia-exposed ARPE-19 cells determined by Western blot analysis; ^∗^*p* < 0.05, compared with control ARPE-19 cells. (g) The protein expression of SOX9 in hypoxia-exposed ARPE-19 cells after different transfection determined by Western blot analysis. (h) Binding sites between SOX9 and LCN2 determined by ChIP-PCR; ^∗^*p* < 0.05, compared with IgG. (i) The effect of SOX9 on LCN2 promoter activity in HEK-293T cells determined by dual luciferase reporter gene assay; ^∗^*p* < 0.05, compared with HEK-293T cells transfected with oe-NC. (j) The protein expression of LCN2 in hypoxia-exposed ARPE-19 cells after different transfection determined by Western blot analysis. The experiment was repeated three times. ^∗^*p* < 0.05 and^∗∗^*p* < 0.01, compared with hypoxia-exposed ARPE-19 transfected with sh-NC; ^#^*p* < 0.05, compared with hypoxia-exposed ARPE-19 cells transfected with oe-NC. ^∗∗∗^*p* < 0.001 and^∗∗∗∗^*p* < 0.0001. ^###^*p* < 0.001.

The article "Sirtuin 1 Induces Choroidal Neovascularization and Triggers Age-Related Macular Degeneration by Promoting LCN2 through SOX9 Deacetylation" was retracted in 2024. Reasons: signs of a paper mill; compromised peer review; unreliable results or conclusions.

**Figure 3:** SIRT1 promotes the SOX9 nuclear translocation through the deacetylation of SOX9, thereby increasing the expression of LCN2. (a) The protein expression of SIRT1 in control and hypoxia-exposed ARPE-19 cells determined by Western blot analysis. ^∗∗^*p* < 0.01, compared with control ARPE-19 cells. (b) The protein of SIRT1 in hypoxia-exposed ARPE-19 cells after different transfection determined by Western blot analysis. ^∗∗∗^ *p* < 0.001 and^∗∗∗∗^*p* < 0.0001, compared with hypoxia-exposed ARPE-19 cells transfected with sh-NC. (c) The protein expression of SOX9 and acetylated SOX9 in hypoxia-exposed ARPE-19 cells after different transfection determined by Western blot analysis. ^∗∗^*p* < 0.01, compared with hypoxia-exposed ARPE-19 cells transfected with oe-NC. ^####^*p* < 0.0001, compared with hypoxia-exposed ARPE-19 cells transfected with sh-NC. (d) The nuclear localization of SOX9 in hypoxia-exposed ARPE-19 cells after different transfections determined by immunofluorescence staining (scale bar: 25 *μ*m). (e) The protein expression of SIRT, acetylated SOX9, and LCN2 in the hypoxia-exposed ARPE-19 cells after different transfections determined by Western blot analysis. (f) The content of VEGF, TNF-*α*, and IL-6 in the conditioned medium of hypoxia-exposed ARPE-19 cells after different transfections determined by ELISA. (g) Hypoxia-exposed ARPE-19 cell viability detected by CCK-8. (h) Hypoxia-exposed ARPE-19 cell apoptosis detected by flow cytometry. (i) HUVEC migration detected by Transwell assay. (j) HUVEC angiogenesis detected by tube formation experiment. In (e)–(h), ^∗^*p* < 0.05, compared with hypoxia-exposed ARPE-19 cells transfected with sh-NC+oe-NC. ^#^*p* < 0.05, compared with hypoxia-exposed ARPE-19 cells transfected with sh-SIRT1+oe-NC. In (i) and (j), ^∗^*p* < 0.05, compared with HUVECs transfected with sh-NC+oe-NC; ^#^*p* < 0.05, compared with HUVECs transfected with sh-SIRT1+oe-NC. ^∗∗^*p* < 0.01,  ^∗∗∗^*p* < 0.001, and^∗∗∗∗^*p* < 0.0001. ^##^*p* < 0.01,  ^###^*p* < 0.001, and^####^*p* < 0.0001.

The article "Sirtuin 1 Induces Choroidal Neovascularization and Triggers Age-Related Macular Degeneration by Promoting LCN2 through SOX9 Deacetylation" was retracted in 2024. Reasons: signs of a paper mill; compromised peer review; unreliable results or conclusions.

**Figure 4:** SIRT1 increases the expression of LCN2 by deacetylating SOX9 to promote the formation of laser-induced CNV in mice. (a) The protein expression of SIRT1, acetylated SOX9, and LCN2 in choroid/RPE tissues of mice determined by Western blot analysis. (b) The protein expression of SIRT1, acetylated SOX9, and LCN2 in choroid/RPE tissues of mice after different treatment determined by Western blot analysis. (c), Immunofluorescence staining analysis of mouse choroid/RPE tissues. Green indicates isolectin B4 and CNV area is within the red line. (d) CNV damage area statistics; scale bar: 50 *μ*m. ^∗^*p* < 0.05, compared with control or mice treated by sh-NC+oe-NC; ^#^*p* < 0.05, compared with mice treated by sh-SIRT1+oe-NC. ^∗∗∗^ *p* < 0.001 and^∗∗∗∗^*p* < 0.0001. ^####^*p* < 0.0001. Measurement data were expressed as the mean ± standard deviation.

**Figure 5:** RGDS inhibited the formation of laser-induced CNV in mice. (a) The protein expression of LCN2 in the choroid/RPE tissues of mice determined by Western blot analysis. (b) The expression of isolectin B4 in the choroid/RPE tissues of mice after different treatments determined by immunofluorescence staining; scale bar: 25 *μ*m. (c) Statistics of CNV damage area. ^∗∗∗∗^*p* < 0.0001 compared with control; ^####^*p* < 0.0001 compared with mice treated by Laser+RGES.

**Figure 6:** Schematic diagram of the mechanism by which SIRT1 influences the formation of CNV caused by AMD. SIRT1 upregulates the expression of LCN2 by deacetylating SOX9 to promote the formation of CNV caused by AMD.

## Data Availability

The data used to support the findings of this study are included within the supplementary information file(s).

## Additional Points

*Data Sharing Statement*. The datasets generated/analysed during the current study are available.

## Supplementary Materials

Supplementary Materials Supplementary Materials Fig. S1: Western blot analysis of E-cadherin, N-cadherin, Snail, and Vimentin proteins in ARPE-19 cells exposed to hypoxia.
